The article "Multiclassification of Endoscopic Colonoscopy Images Based on Deep Transfer Learning" was published in 2021. Journal: Comput Math Methods Med.

# Multiclassification of Endoscopic Colonoscopy Images Based on Deep Transfer Learning

**DOI:** 10.1155/2021/2485934

**Published:** 2021-07-03

**Authors:** Yan Wang, Zixuan Feng, Liping Song, Xiangbin Liu, Shuai Liu

**Affiliations:** ^1^Department of General Surgery, China-Japan Union Hospital of Jilin University, Changchun 130033, China; ^2^Department of Pharmaceutics, College of Pharmacy, Shenyang Pharmaceutical University, Shenyang 110116, China; ^3^College of Computer Science and Technology, Jilin University, Changchun 130012, China; ^4^College of Information Science and Engineering, Hunan Normal University, Changsha 410081, China; ^5^Hunan Xiangjiang Artificial Intelligence Academy, Changsha 410081, China

## Abstract

With the continuous improvement of human living standards, dietary habits are constantly changing, which brings various bowel problems. Among them, the morbidity and mortality rates of colorectal cancer have maintained a significant upward trend. In recent years, the application of deep learning in the medical field has become increasingly spread aboard and deep. In a colonoscopy, Artificial Intelligence based on deep learning is mainly used to assist in the detection of colorectal polyps and the classification of colorectal lesions. But when it comes to classification, it can lead to confusion between polyps and other diseases. In order to accurately diagnose various diseases in the intestines and improve the classification accuracy of polyps, this work proposes a multiclassification method for medical colonoscopy images based on deep learning, which mainly classifies the four conditions of polyps, inflammation, tumor, and normal. In view of the relatively small number of data sets, the network firstly trained by transfer learning on ImageNet was used as the pretraining model, and the prior knowledge learned from the source domain learning task was applied to the classification task about intestinal illnesses. Then, we fine-tune the model to make it more suitable for the task of intestinal classification by our data sets. Finally, the model is applied to the multiclassification of medical colonoscopy images. Experimental results show that the method in this work can significantly improve the recognition rate of polyps while ensuring the classification accuracy of other categories, so as to assist the doctor in the diagnosis of surgical resection.

## 1. Introduction

Image classification is a task that classifies images into a certain category according to different features in the image. It is the core of computer vision to distinguish different categories of images. Image classification is the basis of other high-level visual tasks in computer vision, such as target detection, image segmentation, and face recognition. Image classification is widely used in many fields, such as payment method for face recognition, toll system for license plate recognition, autonomous driving for traffic safety, and computer-aided system for diagnosis [1]. In the medical world, the number of medical images generated every day is uncountable, and a tomographic slice of the lungs of a patient can generate dozens of CT images [2]. Therefore, classifying massive medical images is an important step of computer-aided diagnosis [3, 4].

The article "Multiclassification of Endoscopic Colonoscopy Images Based on Deep Transfer Learning" was published in 2021. Journal: Comput Math Methods Med.

Medical image classification refers to taking one or more examination images as input, predicting them through the trained model, and outputting a diagnostic result indicating whether a certain disease is suffering or whether the severity is graded. At present, it has been widely used in epidemic prevention and diagnosis of benign tumors and cancer and to distinguish between different categories of the same disease and other important clinical events [5]. The object of medical image classification is the image obtained by patients through various kinds of examination equipment, mainly including Computed Tomography (CT), X-ray, Magnetic Resonance Imaging (MRI), and ultrasound image (UI) [6]. In addition, there are other pathological images as well as endoscopic images. When a doctor examines disease in the intestine, the patient generally needs an endoscope to obtain the surface features of the intestine tract to make a diagnosis. The main manifestations of various lesions in the intestine are polyps, inflammation, and cancer. Polyps are spherical or oval pedicled masses protruding from the mucosal surface of the large intestine. It is a common benign tumor. Inflammation is manifested as colonic mucosa with extensive hyperemia, edema, and erosion under a colonoscopy, and it is easy to bleed when touched, with pus and blood and exudate on the surface. Cancer is a common malignant tumor in the gastrointestinal tract. Cancer protrudes into the intestinal lumen and has hemorrhage and necrosis on the surface. The classification of medical colonoscopy images is mainly divided into four categories: polyps, inflammations, cancer, and normal [7].

The research of image classification technology has always attracted attention. In recent years, lots of advanced intelligent classification methods have emerged, and classification accuracy has been continuously improved. However, there are still many problems to be further studied, such as the difficulty of classification and recognition caused by image quality and the inapplicability of feature extraction methods to different images. Traditional medical image classification methods are mainly based on the neural network, Bayesian network, decision tree, and other single modes. With the development of Artificial Intelligence (AI) and the demand for application in the medical field, deep learning has become the mainstream image classification framework. Deep learning simulates the human brain for analytical learning and uses human brain mechanisms to interpret data. Convolutional neural networks (CNN) are the most commonly used network model for deep learning. It sends images into the network for training and classifies image data according to image features. Deep learning requires a large number of data sets to achieve better classification results when training network structures, so as to prevent model overfitting. Due to the complexity and inconvenience of endoscopy, the requirements for doctors and patients in the process of examination are extremely high, which leads to difficulty in the collection of colonoscopy data sets. Aiming at the problem of model overfitting caused by the small amount of colonoscopy images trained by deep learning, this work proposes the use of transfer learning to solve the problem of deep network training requiring a large number of data sets. The contributions of this paper are as follows:

1. Four-classification tasks of the intestinal image are proposed. In order to accurately distinguish all kinds of pathologically similar lesions in the intestinal tract, while improving the classification accuracy of polyps, the colonoscopy images are divided into four categories: normal, polyp, inflammation, and cancer, which increased the diversity of disease types in the classification task
2. Transfer learning is proposed to optimize classical deep learning, and a multiclassification model of endoscopic colonoscopy images based on deep transfer learning was obtained. The pretrained network model on the natural image is used to fine-tune its network with the intestinal image to solve the problem that deep learning training requires a large number of data sets
3. Finally, the feasibility of the proposed method was verified by experiments. Inputting the intestinal image into the model proposed in this paper, four classification results were obtained, which significantly improved the polyp recognition rate while ensuring the classification accuracy of other categories

The following is the structure of this paper. In Section 2, deep transfer learning and intestinal image classification tasks are discussed.  Section 3 introduces the intestinal data set and its classification methods used in this work. In Section 4, the classification methods mentioned are experimented and compared.  Section 5 summarizes the work of this paper and looks forward to future work.

The article "Multiclassification of Endoscopic Colonoscopy Images Based on Deep Transfer Learning" was published in 2021. Journal: Comput Math Methods Med.

## 2. Related Work

### 2.1. Medical Image Classification

Medical image classification is the first major contribution made by deep learning in the field of medical image processing. Medical image processing initially focused on unsupervised pretraining and network structures, such as Stacked Autoencoder (SAES) and Deep Belief Networks (RBMS). As early as 2013, Suk et al. [8] proposed a feature representation and stacked autoencoder based on deep learning, which combined potential information with original low-level features and improved the classification accuracy of Alzheimer's disease (AD)/Mild Cognitive Impairment (MCI). With the rise of large-scale visual recognition challenges such as ImageNet, several excellent deep neural networks have emerged, which promote the development of deep learning. At present, CNN has always been the current standard technology in medical image classification. The pretraining of CNN on natural images has shown amazing results, challenging the authority of human experts in certain classification tasks. Many researchers use classic deep learning networks to improve classification accuracy. For example, Gao et al. [9], in order to grade and evaluate the severity of nuclear cataract, first clustered the images to obtain local filters, then sent the learned filters to the convolutional neural network and recursive neural network for further feature extraction, and finally used Support Vector Machine (SVM) for classification. The results verify that the model is superior to the latest progress in clinical cataract classification. Jiao et al. [10] proposed a breast mass classification framework based on deep features to solve the problem of poor performance of the underlying features. The framework mainly includes a convolutional neural network and a decision mechanism, which combines enhanced information and deep features to simulate the process of doctor diagnosis to improve classification accuracy. Lin et al. [11] proposed a recurrent neural network with an attention model for sequence labeling; in this test, a hierarchical structure to incorporate character-level and word-level information is proposed by applying an attention mechanism to both levels, and the experiment proves its effectiveness. Since generative adversarial networks (GAN) were proposed by Goodfellow and others in 2014, it has occupied a large part of the deep learning network framework and is one of the most promising methods for unsupervised learning on complex distributions in recent years. GAN is composed of two models, generator and discriminator, and the two models play with each other to produce relatively good output [12]. The application of GAN in the field of medical image processing not only is limited to medical image classification but also has a great contribution to segmentation, detection, and enhancement of medical images. In the field of classification, Madani et al. [13] used the semisupervised learning characteristics of the generative adversarial networks. First, the authors solved the problems of medical labeling data scarcity and data overfitting and then used the deep generative adversarial network to learn the vision of the chest X-ray structure to classify abnormal and normal samples. Frid-Adar et al. [14] proposed a network for the classification of liver diseases. First, classical data enhancement is used to enlarge the data sets, and then, GAN technology is used to further expand the size and diversity of the data. Finally, 182 CT images of liver lesions are used for verification, and the sensitivity and specificity of the network are improved after adding synthetic data enhancement. Ma et al. [15] proposed a blood cell image classification framework based on Deep Convolutional Generative Adversarial Network (DC-GAN) and Residual Network (ResNet).

The article "Multiclassification of Endoscopic Colonoscopy Images Based on Deep Transfer Learning" was published in 2021. Journal: Comput Math Methods Med.

### 2.2. Deep Learning

As one of the most cutting-edge scientific and technological fields, deep learning has always been leading the progress of science and technology. It simulates the mechanism of the human brain to interpret data and establish a neural network for analytical learning. With the advent of the era of AI, deep learning has begun to shine in the field of machine learning research and application. The most notable applications are the fields of computer vision and natural language processing [16, 17], implemented by CNN, GAN, and RNN, respectively. Lecun et al. invented CNN as early as the 1990s. With the success of the ImageNet competition, more and more researchers have turned their attention to CNN [18]. Krizhevsky et al. [19], the champion of the ImageNet competition in 2012, first used the ReLU activation function, local response normalization, Dropout, and other tricks; improve the generalization ability of the network; and avoid overfitting of the model. Subsequently, Simonyan and Zisserman [20] proposed VGG, which is improved on the basis of AlexNet. The entire network uses the same size of 3 × 3 convolution kernel, which simplifies the structure of the neural network. In addition, VGG increases the number of layers of convolution since increasing network depth can improve network performance. GoogLeNet continues this feature. In order to prevent problems such as gradient disappearance and overfitting caused by deepening the number of network layers, the authors introduced the Inception structure. Inception improves the training results from another perspective and can extract more features with the same amount of calculation, thereby improving the training results [21]. In order to solve the problem of the inability to train when the level is deepened, He et al. [22] proposed ResNet. The authors use the residual block to learn the representation of the residual between input and output, and the internal residual block uses shortcut connections, which alleviate the problem of gradient disappearance caused by increasing depth in the deep neural network. Huang et al. [23] proposed Densenet in 2017. Inspired by ResNet and Highway Networks, the authors transmit information through a direct connection with a later layer. Its core idea is to establish the connection relationship between different layers, make full use of the characteristics of the image, and further alleviate the problem of gradient disappearance. The recurrent neural network (RNN) is one of the most common deep learning algorithms; it has taken the whole world by storm. Almost all state-of-the-art performance in natural language processing or understanding is attributed to variants of RNN [24].

The article "Multiclassification of Endoscopic Colonoscopy Images Based on Deep Transfer Learning" was published in 2021. Journal: Comput Math Methods Med.

### 2.3. Transfer Learning

Most tasks in medical image processing require doctors to annotate the original image, namely, GroundTruth. Labeling data is a tedious and expensive task. Since medical data is related to the privacy of patients, it is more difficult to build medical data sets. As one of the most effective methodologies in the current deep learning field, transfer learning alleviates the above problems. Transfer learning utilizes the similarity between data, tasks, and models to apply models trained on natural image classification tasks to medical image classification [25].

Long et al. [26] proposed a new adaptive method for the deep network domain, which can jointly learn adaptive classifiers and transferable features from labeled data in the source domain and unlabeled data in the target domain. By inserting several layers in the deep network to learn the residual function of the reference target classifier, classifier adaptation was realized. Chang et al. [27] proposed a multiscale convolutional sparse coding (MSCSC) method with unsupervised transfer learning ability. By strengthening scale specificity and combining automatic learning filter banks at different scales, the basic knowledge of transferability can be learned, and finally, the target task can be fine-tuned. Aiming at the problem of poor application of deep learning in the diagnosis and treatment of multiple retinal lesions, Choi et al. [28] adopted the random forest migration learning method based on the VGG19 structure. The authors found that transfer learning combined with ensemble classifiers can improve classification performance to detect multiclassification retinal diseases. Kaur and Gandhi [29] discussed the ability of the pretrained model DCNN VGG16 with transfer learning ability to classify pathological brain images and replaced the last few layers of the VGG16 model to adapt to new images in current applications. The verification on the test set showed good results in sensitivity, specificity, and accuracy. Hosny et al. [30] proposed a high-performance automatic skin lesion classification system using transfer learning and pretrained deep neural network, AlexNet. The transfer learning is achieved by fine-tuning the weight of the architecture and replacing the classification layer with the softmax layer. Talo et al. [31] proposed deep transfer learning based on ResNet34 to automatically classify normal and abnormal brain MRI images. The authors use data augmentation, optimal-learning rate finder, and fine-tuning to train the model. The model obtained 100% of 5 times classification accuracy on 613 MR images, helping radiologists to perform daily MR imaging examinations.

The article "Multiclassification of Endoscopic Colonoscopy Images Based on Deep Transfer Learning" was published in 2021. Journal: Comput Math Methods Med.

## 3. Materials and Methods

### 3.1. Materials

Compared with other medical data sets, colonoscopy images are more difficult to collect, mainly due to the complexity and inconvenience of the inspection method. Endoscopy is shown in the form of video, and colonoscopy data sets must be viewed from beginning to end to capture frames with key information. The popular medical images of enteroscopy mainly include the Kvasir-SEG intestinal polyp data set (https://www.simula.no/publications/kvasir-seg-segmented-polyp-dataset) [32], CRCHisto Phenotypes datasets (https://warwick.ac.uk/fac/cross_fac/tia/data/crchistolabelednucleihe) [33], and CVC-Clinic data sets (http://www.cvc.uab.es/CVC-Colon/index.php/databases/) [34]. Most of these data sets are used for image segmentation, including intestinal diseases mainly polyps and tumors, and the data types are relatively single.

The experimental data in this paper are from real cases of patients in the anorectal department of a hospital. The colonoscopy images of patients were obtained by endoscopy. First, screening took place to eliminate the unusable data caused by insufficient bowel preparation and the examination process, then data cleaning; finally, a small data set is constructed. The data sets collected 430 intestinal images of patients suffering from various diseases, which are mainly divided into four categories: normal, inflammation, polyps, and cancer. Among them, there are 120 colonoscopy images for normal, 110 colonoscopy images for inflammation, 108 colonoscopy images for polyps, and 92 colonoscopy images for tumors. The category label of each image was obtained by the joint diagnosis of the doctors in the anorectal department, and the subdivided category and characteristics were discussed to obtain the final data sets with the label.  Figure 1 is an example diagram of these data sets.

The article "Multiclassification of Endoscopic Colonoscopy Images Based on Deep Transfer Learning" was published in 2021. Journal: Comput Math Methods Med.

In addition, we have enhanced the data set to increase the diversity of samples, which also made the trained deep learning framework have high generalization ability and strong robustness. Through the four data enhancement methods of brightness enhancement, contrast enhancement, image flip, and angle rotation, 480 images of normal category, 440 images of inflammation category, 432 images of polyp category, and 368 images of tumor category were obtained, respectively.  Figure 2 is the result of data enhancement after randomly selecting one of the images. We randomly select 80% of the pictures from the data set as the training set for training and 20% of the pictures as the test set for testing. The distribution structure is shown in Table 1.

### 3.2. Methods

#### 3.2.1. Multiclassification Task Based on Transfer Learning

Transfer learning refers to the process of knowledge transfer in two different domains. The knowledge learned in the source domain *S* is used to help the learning task in the target domain *T*, and the number of training samples in the source domain is generally far greater than that in the target domain. Generally speaking, according to different ways of transfer, transfer learning is divided into inductive transfer learning and transduction transfer learning. This paper uses inductive transfer learning [35]. The specific implementation ideas are summarized as follows: Firstly, a pretraining model with good generalization performance is obtained by training the deep learning model on the large-scale image classification data set, ImageNet 1000. Then, inductive transfer learning was used to transfer these pretraining models to the intestinal multiclassification model to reduce the training burden of insufficient colonoscopy images in our task. Finally, the model was adjusted and updated by using the established colonoscopy four-classification images to improve the classification accuracy.

*(1) Pretraining Model Processing*. The classic classification deep learning model is used as the classification backbone network to generate the corresponding pretraining model. The essence of generating the pretraining model is to train the data set of the source domain from the beginning using the classification network model. For different layers of CNN, the image features learned by each layer are different. The features learned in the shallower layer are more general, and the features learned in the deeper layer are more relevant to specific tasks. In Figure 3, the shallowest common feature “lines” are the same for the classification task of faces, cars, elephants, and chairs [36]. ImageNet 1000 classification is a subset of ImageNet, with a training set of about 1.2 million pieces, a verification set of 50,000 pieces, and a test set of 100,000 pieces. It belongs to 1,000 different categories, and each image is strictly manually screened and labeled. Multiclassification of a variety of images is implemented on the ImageNet data set, which is more suitable for the target task of this paper. Therefore, we chose to use the model trained on ImageNet 1000 classification to save it as a pretraining model.

*(2) Transfer the Pretraining Model*. The pretraining model used in this paper is a deep neural network, in which the mobility of each layer is not the same. In general, the lower layers of the network learn some general low-level features, the middle or higher layers learn abstract high-level semantic features, and the last layers generally learn task-specific features. Therefore, according to the feature of the target task and its relevance to the source domain, different layers of the pretraining model can be selected to transfer to the target task. In network training, the initial weight and bias of the convolutional layer are randomly assigned, and the quality of this value directly affects the final performance of the model to a large extent. Therefore, we give the convolutional layer an initial weight and bias and then continuously adjust to the task itself based on the feedback of the network. In this paper, the convolutional layer of other pretrained models is transferred to the colonoscopy image classification task, and the fully connected layer is retrained.

*(3) Fine-Tuning*. Fine-tuning is essential for a successful deep transfer learning model. The parameters of the pretraining model were adjusted by the similarity of the data between the pretrained data set and the colonoscopy image data set. During this process, we made several attempts. As shown in Figure 4, the ImageNet 1000 classification model is on the left and the colonoscopy classification model is on the right. In this paper, the weight and bias of the initial convolutional layer of the pretraining model remain unchanged, and only the fully connected layer related to the final output classification result is modified. The training model was adjusted by using the four-classification data of colonoscopy to find an optimal parameter of the full connective layer. Finally, according to the classification results, the best match between the convolutional layer and the fully connected layer is found, and the best parameters of the fully connected layer are saved to obtain an optimal complete model.

The article "Multiclassification of Endoscopic Colonoscopy Images Based on Deep Transfer Learning" was published in 2021. Journal: Comput Math Methods Med.

#### 3.2.2. Deep Learning Model Based on Transfer Learning

The mainstream deep learning model in medical image classification tasks is mainly CNN. Since the development of CNN, there have been many types of excellent network frameworks. Among them, several classic models have milestone significance in the development of CNN, such as LeNet, AlexNet, VGG, and GoogLeNet. For the data sets and tasks used in this paper, we choose AlexNet, VGG, and ResNet as the backbone network from the depth of the network. This section discusses the deep convolutional network we use based on transfer learning.

The AlexNet network itself uses many modern deep convolutional network technical methods, and its network structure is shown in Figure 5. It uses Dropout to alleviate the occurrence of overfitting problems and make the model more generalized. The GPU is used for parallel training, so that the model can be trained quickly. In addition, AlexNet amplifies the data set by making small changes to the original image and uses data enhancement to improve the accuracy of the model. Therefore, AlexNet embodies unique advantages in solving large-scale data classification problems [19]. We used AlexNet for the transfer learning of ImageNet 1000 classification, and the AlexNet parameters trained by ImageNet were transferred to the intestinal image training task. When initializing the convolutional layers of the first five layers, the existing parameters are used, while random initialization is used in the full connection layer of the last three layers, and then, adjustments are made according to the intestinal data set.

According to the size of the established data set, AlexNet is beneficial to improve classification accuracy. In addition, AlexNet uses ReLU as the activation function to solve the situation where the gradient disappears when the Sigmoid function is backpropagated, which is conducive to the training of the model. The formula is as follows:

(1) $$\begin{array}{c} f\left(x\right)=\max\left(0,x\right). \end{array}$$

When VGG is used for large-scale image classification, it can be extended to various tasks and data sets. According to the characteristics of our task, VGG, which is suitable for arbitrary classification, is applied to the four classifications of intestinal image. VGG emphasizes the depth in the design of convolutional neural networks, and the accuracy of ImageNet 1000 classification is also different for different network depths. VGG uses a smaller convolution kernel to replace a large-size convolution, which saves computing resources, thereby setting aside resources for deepening the network. There are 5 convolutions in VGG; each convolutional layer is followed by a pooling layer. The network structure is shown below. The expansion performance of its network is more prominent; there are mainly two commonly used layers, VGG16 and VGG19. We use VGG16 and VGG19 to set an initial value for the convolution layer in the two models by training on ImageNet 1000 classification and do not deal with other layers. The concise structure of VGG16 and VGG19 makes its migration performance good, and the process of migrating to other data sets is simple [20].

The article "Multiclassification of Endoscopic Colonoscopy Images Based on Deep Transfer Learning" was published in 2021. Journal: Comput Math Methods Med.

Considering that the gradient disappears more obviously with the increase in the number of layers of the neural network during the training of intestinal image, we considered using ResNet with a residual structure to obtain better results [22]. ResNet was trained by using ImageNet, the pretraining data set we selected. Since its network is no longer a simple stacked structure, it solves the problem of less and less obvious gradients caused by the increase in the number of network layers. The formula is defined as follows:

(2) $$\begin{array}{c} y=F\left(x,\left\{w_{i}\right\}\right)+x, \end{array}$$

where *x* and *y* are the input and output vectors of this layer. The *F*(*x*, {*w*_*i*_}) function represents the remaining mappings to be learned. The obtained ResNet pretraining model solves the problems of information loss and loss to some extent. By directly passing the input information to the output, the integrity of the information is protected and the learning objectives and difficulty are simplified.

## 4. Experimental Results and Analysis

In this section, we discuss the results obtained when the proposed multiclassification method based on deep transfer learning is applied to the proposed colonoscopy image data set. In order to prove that our proposed method is feasible, we selected multiple commonly used deep learning networks to compare the performance of each network. The parameter setting of the experiment is introduced in detail below, and results of the experiment are analyzed at last.

### 4.1. Setting of Experimental Parameters

This experiment is based on Tensorflow and runs under the Ubuntu 16.04.5 LTS system. The hardware includes AMD Ryzen 5 1600 Six-Core Processor, NVIDIA GeForce GTX 1080 GPU.

1. *Size Selection*. The size of the data set is not uniform. The average width, maximum width, and minimum width are 780, 886, and 750, respectively. The average height, maximum height, and minimum height are 655, 729, and 599, respectively. The original shape of the intestinal wall will be destroyed after cutting from the colonoscopy image. However, without cutting, the size of the colonoscopy image cannot be unified, and it is difficult to use deep learning for classification learning. Considering that the background of colonoscopy images is a mostly round-like intestinal wall, the original image size is changed to a size of 224 × 224 through the resize operation. The bit depth of the image is uniformly modified to 24. In order to maintain the integrity of the intestinal wall in the image while making the data meet the input requirements of the model in this paper, we unified the data size to 224 × 224 × 3.
2. *Function Selection*. As a classic loss function in classification tasks, cross-entropy can avoid gradient dispersion when performing gradient descent calculations, resulting in a decrease in the learning rate. It makes the learned model distribution closer to the real data distribution, thereby improving the accuracy of multiclassification. ReLU is selected as the activation function. Compared with Sigmoid and Tanh, the actual convergence speed is faster and there is no complex exponential operation, which makes the network training faster. After comparing several optimization functions: ADAM, RMSProp, and SGD, we finally choose SGD as our optimization function.
3. *Migration Layer Selection*. Considering that all the layer features in the original task do not promote the target task, only partial layer migration is carried out. We choose to use all the convolutional layer parameters obtained on the pretrained model to train the fully connected layer in the target domain after migration.
4. *The Other*. During model training, the batch size was 64, the epoch was equal to 10000, and the learning rate was set to 0.0001.

The article "Multiclassification of Endoscopic Colonoscopy Images Based on Deep Transfer Learning" was published in 2021. Journal: Comput Math Methods Med.

### 4.2. Analysis of Experimental Results

To demonstrate the effectiveness of our proposed model, we evaluated the performance of the target model through repeated validation. We divide the experiment into four groups, do not add transfer learning and data enhancement, add data enhancement without transfer learning, only add transfer learning without data enhancement, add transfer learning and data enhancement, and compare and analyze the impact of each strategy on accuracy. The classic deep learning models used in the experiment include AlexNet, VGG16, VGG19, ResNet50, and ResNet101.

In this experiment, we compared the classification accuracy of the traditional deep learning model and the proposed solution. The experimental results obtained are as follows. The models proposed in this paper have better performance than traditional deep learning models.

First of all, we trained each classical deep learning model from beginning to end to apply the four classifications of colonoscopy images without any data enhancement and transfer learning in the textual colonoscopy data set. Secondly, in order to compare the effect of transfer learning, we used the model of transfer learning training to get another set of results. Due to the small amount of data, if the data set is divided into 8 training sets and 2 test sets, the experimental results show that the model is easy to overfit. Therefore, 90% of the 430 data sets were randomly selected in this paper as the training set and 10% as the test set, and the results are obtained as shown in Tables 2 and 3, respectively. Tables 2 and 3 describe the number and accuracy of the correct classification of the four categories on each model, where *T* represents that the actual category is identical to the predicted category.

On the basis of data enhancement of the data set, we use the multiclassification model based on deep transfer learning proposed in this paper for training. By comparing the data enhancement strategy training model and the transfer learning combined with the data enhancement strategy training model, the effectiveness of transfer learning is verified. Since the amount of data has increased after data enhancement, this paper divides the data set according to 8 : 2 of the training set to the test set. The results shown in Tables 4 and 5 were obtained, respectively.

The experimental results under the two models are compared, as shown in Table 6. Due to the small number of data sets and the difference in the number of classifications from the widely used diconomies in the conventional models, the classification effect of the traditional deep learning model is poor. In the same data set, it can be seen that accuracy of the model using transfer learning is greatly improved compared with the traditional deep learning model.

Deep learning requires a large number of data sets for training to prevent overfitting of the model, and such a large amount of data is more beneficial to transfer learning. Suppose the sample space of a machine learning task *T* is *x* × *y*, where *x* is the input space and *y* is the output space, and its probability density function is *p*(*x*, *y*). Learn from the statistical point of view; a machine learning task *T* is defined as a modeling problem of conditional probability *p*(*y*  |  *x*) in a domain *D*.  Table 7 shows a comparison between transfer learning and standard machine learning. Therefore, the results of transfer learning are better than traditional deep learning models.

The article "Multiclassification of Endoscopic Colonoscopy Images Based on Deep Transfer Learning" was published in 2021. Journal: Comput Math Methods Med.

We output the confusion matrix of the four classification results of each model in the intestine, as shown in Figure 6. Among them, 0 represents cancer, 1 represents inflammation, 2 represents normal, and 3 represents polyps. Among the five transfer learning models, ResNet50-tl has the best performance compared with the other models, with a performance of 94.48%. ResNet50 improves the accuracy of the network by using residuals to deepen the network structure. VGG only increases the depth of the network by simply superimposing the convolutional layer, which leads to the disappearance of the model gradient; thus, the classification accuracy is not high. Compared with the scale of the data set used in this paper, ResNet101 has too many layers in the network, which easily leads to overfitting of the model. Among the four types of colonoscopy images, polyps were correctly diagnosed more often than the other two types of diseases except for normal types. The characteristics of polyp lesions are outstanding, and feature extraction is used. Under the condition of ensuring the classification accuracy of other categories, the model can improve the number of polyp diagnosis and assist doctors in making judgments. Therefore, it is confirmed through experiments that the ResNet four-classification of intestines based on transfer learning alleviates the problem of small data sets in medical image processing. Transfer learning makes the model more robust and generalizable, which is of great clinical value.

## 5. Conclusion and Prospect

At present, with the continuous improvement of medical technology, computer-aided diagnosis has occupied an important position in the medical industry. In particular, the combination of deep learning and medical image processing has been deeply explored by many researchers. In this interdisciplinary field of integrated medical imaging, mathematical modeling, digital image processing, and so on, there are still many complex and diverse problems that need to be solved urgently.

In medical image analysis, the cost of data acquisition and annotation is high, and it is very difficult to construct a large-scale standard data set, which hinders the development of medical image diagnosis. The common solution is to use data enhancement techniques common in deep learning, such as geometric transformation and color transformation. This paper proposes a deep learning framework based on transfer learning for multidisease colonoscopy image classification. The network model with better training results on natural images is transferred to the specified classification task, and the existing data sets are used to fine-tune the tasks. Finally, the feasibility of the proposed method is verified by experiments. Using this method can help us save training time and improve learning accuracy. Generally, pretrained models are trained on a large data set, which invisibly expands our training data sets and makes the model more robust and capable of generalization.

The article "Multiclassification of Endoscopic Colonoscopy Images Based on Deep Transfer Learning" was published in 2021. Journal: Comput Math Methods Med.

With the development of deep learning, deep transfer learning will be widely used to solve many challenging problems. However, transfer learning also has its shortcomings. For example, categories that exist only in the source domain but not in the target domain will have a negative transfer impact on the transfer result. Therefore, we need to go one step further and develop different strategies of transfer learning for the deep network.

## Figures and Tables

**Figure 1:** Sample images of four types of colonoscopy in the data set.

**Figure 2:** The effect of data enhancement.

**Figure 3:** Features learned from different object classes.

**Figure 4:** Schematic diagram of fine-tuning in deep learning.

**Figure 5:** The network structure of AlexNet, VGGNet16, and VGGNet19.

**Figure 6:** Confusion matrix diagram of four classifications of each model.

**Table 1:** Distribution of test and training data.

Data category	Normal	Inflammation	Polyp	Cancer	Total quantity
Number of test sets	120	110	110	95	435
Number of training sets	480	440	430	365	1715
Total quantity	600	550	540	460	2150

**Table 2:** Classification results on the traditional deep learning model.

Model	Normal (*T*/total)	Inflammation (*T*/total)	Polyp (*T*/total)	Cancer (*T*/total)	Accuracy (%)
AlexNet	3/12	5/11	8/11	2/9	41.86
VGG16	10/12	4/11	10/11	8/9	74.42
VGG19	11/12	9/11	7/11	1/9	65.12
ResNet50	11/12	10/11	10/11	5/9	83.72
ResNet101	9/12	9/11	6/11	8/9	74.42

**Table 3:** Classification results on the deep transfer learning model.

Model	Normal (*T*/total)	Inflammation (*T*/total)	Polyp (*T*/total)	Cancer (*T*/total)	Accuracy (%)
AlexNet-tl	6/12	6/11	8/11	4/9	55.81
VGG16-tl	10/12	7/11	10/11	7/9	79.07
VGG19-tl	9/12	8/11	8/11	5/9	69.77
ResNet50-tl	11/12	10/11	10/11	8/9	90.70
ResNet101-tl	10/12	9/11	8/11	8/9	81.40

**Table 4:** Classification results of traditional deep learning model based on data enhancement.

Model	Normal (*T*/total)	Inflammation (*T*/total)	Polyp (*T*/total)	Cancer (*T*/total)	Accuracy (%)
AlexNet	81/120	47/110	69/110	23/95	50.57
VGG16	112/120	67/110	79/110	76/95	76.78
VGG19	101/120	47/110	83/110	61/95	67.13
ResNet50	109/120	97/110	96/110	79/95	87.59
ResNet101	106/120	88/110	90/110	63/95	79.77

**Table 5:** Classification results of deep transfer learning model based on data enhancement.

Model	Normal (*T*/total)	Inflammation (*T*/total)	Polyp (*T*/total)	Cancer (*T*/total)	Accuracy (%)
AlexNet-tl	89/120	56/110	79/110	31/95	58.62
VGG16-tl	119/120	72/110	87/110	82/95	82.76
VGG19-tl	106/120	52/110	91/110	67/95	72.64
ResNet50-tl	115/120	106/110	102/110	88/95	94.48
ResNet101-tl	111/120	95/110	98/110	72/95	86.44

The article "Multiclassification of Endoscopic Colonoscopy Images Based on Deep Transfer Learning" was published in 2021. Journal: Comput Math Methods Med.

**Table 6:** Comparison of classification models on traditional deep learning models and deep transfer-based learning.

Model	AlexNet		VGG16		VGG19		ResNet50		ResNet101	
	Traditional	Our	Traditional	Our	Traditional	Our	Traditional	Our	Traditional	Our
Acc (%)	41.86	55.81	74.42	79.07	65.12	69.77	83.72	90.70	74.42	81.40
Acc-DA (%)	50.57	58.62	76.78	82.76	67.13	72.64	87.59	94.48	79.77	86.44

**Table 7:** Comparison of transfer learning and standard machine learning.

Learning type	Sample space	Probability distribution
Standard machine learning	*x*_*S*_ = *x*_*T*_, *y*_*S*_ = *y*_*T*_,	*p*_*S*_(*x*, *y*) = *p*_*T*_(*x*, *y*)
Transfer learning	*x*_*S*_ ≠ *x*_*T*_ or *y*_*S*_ ≠ *y*_*T*_ or *p*_*S*_(*x*, *y*) ≠ *p*_*T*_(*x*, *y*)	

## Data Availability

The colonoscopy image data used to support the findings of this study are available from the first author upon request.
